The article "HO-1 Contributes to Luteolin-Triggered Ferroptosis in Clear Cell Renal Cell Carcinoma via Increasing the Labile Iron Pool and Promoting Lipid Peroxidation" was published in 2022. Journal: Oxid Med Cell Longev.

# HO-1 Contributes to Luteolin-Triggered Ferroptosis in Clear Cell Renal Cell Carcinoma via Increasing the Labile Iron Pool and Promoting Lipid Peroxidation

**DOI:** 10.1155/2022/3846217

**Published:** 2022-04-25

**Authors:** Shangting Han, Fangyou Lin, Yucheng Qi, Cong Liu, Linxiang Zhou, Yuqi Xia, Kang Chen, Ji Xing, Zilin Liu, Weimin Yu, Yunlong Zhang, Xiangjun Zhou, Ting Rao, Fan Cheng

**Affiliations:** ^1^Department of Urology, Renmin Hospital of Wuhan University, Wuhan 430060, China; ^2^Department of Gastroenterology, Renmin Hospital of Wuhan University, Wuhan 430060, China; ^3^Department of Orthopedics, Renmin Hospital of Wuhan University, Wuhan 430060, China

## Abstract

Ferroptosis, a novel form of regulated cell death characterized by disrupted iron metabolism and the accumulation of lipid peroxides, has exhibited enormous potential in the therapy of cancer particularly clear cell renal cell carcinoma (ccRCC). Luteolin (Lut), a natural flavonoid widely existing in various fruits and vegetables, has been proven to exert potent anticancer activity *in vitro and in vivo*. However, previous studies on the anticancer mechanism of Lut have been shown in apoptosis but not ferroptosis. In the present study, we identified that Lut substantially inhibited the survival of ccRCC *in vitro and in vivo*, and this phenomenon was accompanied by excessively increased intracellular Fe^2+^ and abnormal depletion of GSH. In addition, Lut induced the imbalance of mitochondrial membrane potential, classical morphological alterations of mitochondrial ferroptosis, generation of ROS, and occurrence of lipid peroxidation in an iron-dependent manner in ccRCC cells. However, these alterations induced by Lut could be reversed to some extent by the iron ion chelator deferiprone or the ferroptosis inhibitor ferrostatin-1, indicating that ccRCC cells treated with Lut underwent ferroptosis. Mechanistically, molecular docking further established that Lut probably promoted the heme degradation and accumulation of labile iron pool (LIP) by excessively upregulating the HO-1 expression, which led to the Fenton reaction, GSH depletion, and lipid peroxidation in ccRCC, whereas blocking this signaling pathway evidently rescued the Lut-induced cell death of ccRCC by inhibiting ferroptosis. Altogether, the current study shows that the natural compound monomer Lut exerted anticancer efficacy by excessively upregulating HO-1 expression and activating LIP to trigger ferroptosis in ccRCC and could be a promising and potent drug candidate for ccRCC treatment.

## 1. Introduction

Renal cell carcinoma (RCC) is a malignant neoplastic disease originating from the proximal tubular epithelium and frequently occurs in male and elderly individuals, and its incidence trends upward annually worldwide [1]. RCC accounts for approximately 80%–90% of adult renal malignancies, and clear cell RCC (ccRCC, also named KIRC) is the most common histologic subtype [2]. Although early-stage and limited renal cancer is curable by radical surgery, the postoperative recurrence rate is still as high as 40% [3–5]. For advanced and metastatic renal cancer, therapeutic options and effectiveness are often limited due to inherent high resistance to conventional chemotherapy, radiotherapy, and hormonal therapy, making this disease one of the most challenging clinical problems in urology [6]. Therefore, new anticancer strategies should be identified, and safe and effective drugs should be developed.

Ferroptosis, which is biochemically and morphologically distinct from traditional forms of cell death (such as apoptosis, necrosis, pyroptosis, and autophagy), is a novel form of regulated cell death characterized by the disorder of iron metabolism and accumulation of lipid peroxides [7]. Ferroptosis has been previously reported to exert an important role in neurodegenerative diseases, ischemic organ damage, and tumor cell death [8, 9]. Therefore, triggering ferroptosis may be a new promising strategy for the treatment of cancers. The kidney performs an important role in the metabolism and homeostasis of iron, and iron metabolism disorders are also closely implicated in the development and progression of many tumors [10, 11]. Encouragingly, a growing number of studies demonstrated that ferroptosis represents a targetable susceptibility and functions as a tumor suppressor by killing cancer cells in ccRCC [12–14]. Thus, the induction of ferroptosis is emerging as a promising therapeutic strategy for the treatment of ccRCC.

Recently, several natural chemical compounds of plant origin, i.e., artemisinin, brucine, erianin, and trigonelline, have been demonstrated to be effective in triggering ferroptosis and killing cancer cells [15–18]. Accordingly, the research and exploitation of natural products to induce ferroptosis in ccRCC are relevant for the clinical treatment of ccRCC. Luteolin (Lut; 3,4,5,7-tetrahydroxy flavone, Figure 1(a)), a natural flavonoid that is extensively available in various fruits and vegetables, has been proven to exert several pharmacological activities, such as killing tumors, ameliorating inflammation, inhibiting fibrosis, and antiviral properties [19–21]. Lut has shown a wide range of antitumor functions through promoting tumor cell death, inhibiting angiogenesis, reducing drug resistance, restraining epithelial-mesenchymal transition, and suppressing cancer cell invasion and metastasis [22].

Heme oxygenase-1 (HO-1), also known as heat shock protein 32, is a phase II enzyme that metabolizes heme to biliverdin, carbon monoxide, and ferrous ion (Fe^2+^) [23]. Traditionally, HO-1 is extensively recognized as a survival factor that exerts cytoprotective defense functions under various stress conditions. However, the latest studies reveal a dark aspect of HO-1 that makes it dual in nature [24, 25]. The activation of HO-1 within normal levels exerts a cytoprotective effect, whereas the excessive activation of HO-1 leads to the massive accumulation of labile iron pool (LIP) and production of reactive oxygen species (ROS) by accelerating heme metabolism. This phenomenon overwhelms the buffering capacity of ferritin and leads to a severe cytotoxic effect, i.e., ferroptosis [26]. For its central position in the metabolism of Fe^2+^, HO-1 has become a crucial candidate in the therapeutic treatment of cancer through the induction of ferroptosis. In addition, TCGA database indicates that the basal expression of HO-1 is active in ccRCC in the routine state and ranks first in pan-cancer, providing the possibility to manipulate its remarkable regulation in ccRCC. Numerous previous studies demonstrated that Lut upregulates the expression of the NRF2/HO-1 axis due to its pharmacological properties, implying that Lut most probably triggers ferroptosis in ccRCC through its activating effect on HO-1 [27, 28]. Consequently, in the present study, we investigate the role and underlying mechanisms of ferroptosis and HO-1 in Lut-induced cell death of ccRCC.

## 2. Materials and Methods

### 2.1. Reagents

Lut (CAS no. 491-70-3), ferrostatin-1 (Fer-1, CAS no. 347174-05-4), deferiprone (DFP, CAS no. 30652-11-0), zinc protoporphyrin (Znpp, CAS no. 15442-64-5), acetylcysteine (NAC, CAS no. 616-91-1), and ammonium iron (III) citrate (FAC, CAS no. 1185-57-5) were purchased from MedChemExpress (Shanghai, China). Erastin (CAS no. S7242) was purchased from SelleckChem Company (Shanghai, China). These compounds were all dissolved in DMSO (final concentration of less than 0.1% (*v*/*v*)).

### 2.2. Cell Culture

Human ccRCC (i.e., 786-O and OS-RC-2) and human renal tubular epithelial (i.e., HK-2) cell lines were purchased from the Cell Bank of the Chinese Academy of Sciences. 786-O and OS-RC-2 cells were cultured in the RPMI-1640 medium (Gibco, Thermo Fisher Scientific, USA) supplemented with 10% fetal bovine serum (FBS; Invitrogen, Thermo Fisher Scientific, USA) and 1% antibiotics (Biosharp, China). HK-2 cells were cultured in DMEM-F12 medium (Gibco, Thermo Fisher Scientific, USA) supplemented with 10% FBS and 1% antibiotics. Cells were maintained at 5% CO_2_ and 37°C in a humid atmosphere.

### 2.3. Cell Viability Assay

Cell viability assays were performed using the Cell Counting Kit-8 assay (Biosharp, China) in 786-O and OS-RC-2 cells to investigate the killing effect and half maximal inhibitory concentration (IC50) of Lut on ccRCC cells. A total of 5 × 10^3^ cells per well (786-O and OS-RC-2) were seeded into 96-well plates and treated with erastin or Lut with or without DFP/Fer-1 for 24 h. Cells were incubated with 10 *μ*l CCK-8 solution per well for 30 min, and absorbance was measured at a wavelength of 450 nm by using an enzyme marker.

### 2.4. Lactate Dehydrogenase (LDH) Release Cell Death Assay

The LDH Cytotoxicity Assay Kit (Beyotime Biotech, China) was used to assess cell death rate in accordance with the instructions. Following the treatment by different reagents for 24 h, the 96-well plate was centrifuged at 400 × *g* for 5 min. The supernatant (120 *μ*l) from each well was collected and added to the corresponding well of a new 96-well plate. The absorbance was measured at 490 nm.

### 2.5. Measurement of Intracellular GSH

Intracellular GSH levels were measured using the GSH Assay Kit (Nanjing Jiancheng Bioengineering Institute, China). Briefly, cells from each treatment group were collected and centrifuged to obtain the supernatant. The working solution was added to the supernatant and then centrifuged at 800 × *g* for 10 min. The mixture (1 ml) was collected for color development reaction in accordance with the instructions. Each treatment group (100 *μ*l) was collected and placed in a 96-well plate, and the absorbance was measured at 420 nm.

### 2.6. Ferrous Ion Assay

Fe^2+^ levels in cells and tissues of each treatment group were specifically determined using the iron assay kit (Abcam, USA) in accordance with the manufacturer's instructions. Free Fe^2+^, rather than Fe^3+^ or Fe^2+^ complexed in heme, reacts specifically with Ferene S to produce a stable colored complex with absorbance at 593 nm. The collected cells and tissues were homogenized following the addition of iron assay buffer. The mixture was centrifuged at 8000 × *g* and 4°C for 15 min. The supernatant (50 *μ*l) was mixed with 100 *μ*l iron probe and incubated for 1 h at 25°C in the dark. The absorbance of each treatment group was measured at 593 nm by using an enzyme marker. A standard curve was established to calculate the Fe^2+^ level of each group.

### 2.7. Heme Assay

The heme content of each sample was measured by using a QuantiChrom Heme Assay Kit (BioAssay Systems, USA) according to the manufacturer's instructions. Briefly, heme was determined using the 96-well plate protocol. The samples were mixed with working reagents and incubated for 5 min at room temperature, and the absorbance of each well was determined at 400 nm with a microplate reader.

### 2.8. Colony Formation Assay

Colony formation assays were performed to investigate the long-term toxicity of Lut on the proliferation of ccRCC cells. 786-O or OS-RC-2 cells (500 cells/well) were seeded into 6-well plates and treated with or without Lut for 14 days, during which the medium was changed once. Following incubation, cells were fixed with 4% paraformaldehyde for 30 min and then stained with 0.1% crystal violet solution for 15 min at room temperature. The 6-well plates with colonies were dried in air at room temperature. The number of colonies was counted under the microscope (Olympus, Japan).

### 2.9. Wound Healing Assay

786-O or OS-RC-2 cells were seeded into 6-well plates at a density of 80%. The cell monolayer was scratched with a sterile 200 *μ*l pipette tip. Each well was washed twice with PBS and incubated with serum-free medium with or without Lut for 24 h. The width of the wound was imaged at 0 and 24 h by using light microscopy (Olympus, Japan), and images were analyzed using the ImageJ software.

### 2.10. Transwell Invasion Assay

Transwell invasion assay was applied to assess the effects of Lut on the invasiveness of ccRCC cells. Transwell chambers (BD Biosciences, USA) were used to assay cell migration ability. 786-O or OS-RC-2 cells (3 × 10^4^ cells/well) were seeded into the upper chamber and cultured in serum-free RPMI medium, and complete medium containing 10% FBS was added to lower chambers. After incubation of the 24-well plates at 37°C for 24 h, the migrated cells in the lower chamber were fixed with 4% paraformaldehyde for 30 min at room temperature and stained with 0.1% crystal violet for 20 min. The migrated cells were washed with PBS and then observed under an orthomosaic microscope (Olympus, Japan).

### 2.11. Transfection of Small Interfering RNA (siRNA)

HO-1 (human, 5′-CGATGGGTCCTTACACTCA-3′) and NC (5′-TTCTCCGAACGTGTCACGTdTdT-3′) siRNA were purchased from RiboBio (Guangzhou, China). The Lipofectamine 2000 transfection reagent was purchased from Invitrogen (Thermo Fisher Scientific, USA). 786-O and OS-RC-2 cells were fused into 70% in 6-well plates within 24 h. HO-1 or scrambled siRNA (5 *μ*l) was mixed with 5 *μ*l Lipofectamine 2000 transfection reagent to prepare the transfection complex. The mixing system was incubated at room temperature for 15 min and then uniformly added to each group of cells for further experiments. The transfection efficiency was determined using the western blot.

### 2.12. Phalloidin Staining

Cells treated with different conditions were fixed with 4% paraformaldehyde for 30 min and washed thrice with PBS for 5 min each and stained with 200 *μ*l phalloidin solution for 40 min at 37°C. The slides were then washed with PBS and stained with DAPI for 5 min at room temperature in the dark. Images were acquired and analyzed using an orthofluorescence microscope (Olympus, Japan).

### 2.13. 5-Ethynyl-2′-deoxyuridine (EdU) Proliferation Assay

The EdU DNA Proliferation and Detection kit (RiboBio, China) was used to visualize the proliferation of cells in each group. The cells of each treatment group in 6-well plates were fixed with 4% paraformaldehyde for 30 min and then incubated with 0.5% Triton X-100 for 10 min. The slides were incubated with 100 *μ*l of 1× Apollo staining reaction solution for 30 min at room temperature in the dark and then permeabilized with 0.5% Triton X-100 2–3 times for 10 min each. Slides were restained with DAPI and then observed using orthofluorescence microscopy.

### 2.14. Total ROS Assay

Cells of different treatment groups were incubated with 5 *μ*M dihydroethidium (DHE, keygenbio, China) for 30 min at 37°C in the dark and washed thrice with PBS for 5 min each time. Finally, cells were stained with DAPI for 10 min in the dark. Images were acquired and analyzed using an orthofluorescence microscope.

### 2.15. Lipid Peroxidation Assessment

Relative lipid reactive oxygen levels in cells were assessed using the C11 BODIPY 581/591 lipid peroxidation fluorescent probe (Maokangbio, MX5211-1MG, China). The cells of each group were incubated with 5 *μ*M C11-BODIPY for 30 min at 37°C. Images were acquired and analyzed using an orthofluorescence microscope. Reduced state dyes were measured with Ex/Em = 581/591 nm (Texas Red filter), and oxidized dyes were measured with Ex/Em = 488/510 nm (FITC filter).

### 2.16. Mitochondrial Membrane Potential Assay

The mitochondrial membrane potential assay kit with JC-1 (Beyotime Biotech, China) was used to detect changes in the mitochondrial membrane potential in accordance with the manufacturer's instructions. Red (excitation wavelength: 525 nm; emission wavelength: 590 nm) and green (excitation wavelength: 490 nm emission wavelength: 530) fluorescent dyes were used to assess JC-1 aggregates and monomer, respectively. The relative proportion of red and green fluorescence was determined as the proportion of mitochondrial depolarization.

### 2.17. Transmission Electron Microscopy

OS-RC-2 cells cultured in 60 mm dishes were treated with or without Lut for 24 h. Cells were then centrifuged at 70 g for 5 min at room temperature to the bottom of the tube to obtain cell clumps, and the culture medium was discarded. The cell clumps were fixed with 2% glutaraldehyde at 4°C for 2–4 h. Cells were rinsed thrice with PBS (pH 7.4) for 15 min each time and fixed with 1% osmium acid-0.1 M phosphate buffer PBS (pH 7.4) at room temperature (20°C) for 2 h. After rinsing with PBS (pH 7.4), cells were sequentially dehydrated in 50%, 70%, 80%, 90%, 95%, 100%, and 100% alcohol for 15 min each time. Ultrathin sections (60–80 nm) were obtained after permeabilization overnight and embedding for 48 h. Finally, sections were stained twice with uranium-lead (2% aqueous uranyl acetate solution-lead citrate) for 15 min each time and dried at room temperature overnight. Sections were observed using transmission electron microscopy, and images were collected for analysis.

### 2.18. Immunofluorescence Staining

Slides containing 786-O cells were fixed with 4% paraformaldehyde and incubated with BSA for 30 min and with the primary antibody HO-1 (1 : 100, ab13243, Abcam, USA) or glutathione peroxidase 4 (GPX4; 1 : 100, ab125066, Abcam, USA) at 4°C overnight. The next day, slices were incubated with appropriate fluorescently labeled IgG for 50 min at room temperature. Nuclei were stained with DAPI for 10 min. Changes in protein expression were observed by fluorescence microscopy, and image acquisition was performed.

### 2.19. Tumor Xenograft Model

Twenty male BALB/c nude mice (age: 4–6 weeks old) were obtained from the Center of Experimental Animals at Wuhan University Medicine College (Hubei, China). Under conditions of free access to food and water, animals were placed in an environment with an artificial 12 h light/dark cycle at 25°C and 50% relative humidity. PBS (100 *μ*l) containing OS-RC-2 cells (5 × 10^6^) was injected subcutaneously into the right side of the back of each mouse. Tumors reached 50–100 mm^3^ after about seven days. Mice were then randomly assigned to five different treatment groups (i.e., NC, Lut (50 mg/kg), erastin (50 mg/kg), Lut+DFP (75 mg/kg), and Lut+Znpp (25 mg/kg)). Mice were treated with the intraperitoneal injection of erastin or Lut in 100 *μ*l vehicle once every two days for seven times. The DFP/Znpp in 100 *μ*l vehicle was injected intraperitoneally into nude mice once a day for seven times prior to Lut administration. Tumor volumes were measured every two days and calculated as follows: (length × width^2^)/2. One day after the last treatment, mice were euthanized. Tumor weights were measured immediately, and tumor tissues were subsequently collected for further studies. All procedures involving mice were performed in accordance with the National Institutes of Health Guide for the Care and Use of Laboratory Animals and approved by the Ethical Committee for Animal Experimentation, Renmin Hospital of Wuhan University.

### 2.20. Malondialdehyde (MDA) Assay

The content of MDA was measured to reflect the degree of lipid peroxidation in tumor tissues, which indirectly indicated the degree of cellular damage. MDA levels in each group of tumor tissues were measured using the MDA kit (Nanjing Jiancheng Bioengineering Institute, China) in accordance with the manufacturer's protocol. For each sample, the MDA content was expressed as the absorbance at 532 nm under a microplate reader. Each group was replicated and measured thrice.

### 2.21. Histology and Immunohistochemistry Assay

Tumor tissue sections with thickness of 5 *μ*m were dewaxed in xylene for 20 min at room temperature, rehydrated in alcohol, and stained with hematoxylin and eosin for histological examination. Slices were then placed in EDTA buffer for microwave repair and treated in 3% H_2_O_2_ for 10 min to inhibit the endogenous peroxidase activity. Slides were incubated with 5% BSA for 20 min and incubated with 5% BSA for 20 min. Then, tissue slices were incubated with primary antibodies HO-1 (1 : 100, ab13243, Abcam, USA), GPX4 (1 : 100, ab125066, Abcam, USA), SLC7A11/XCT (1 : 100, 26864-1-AP, Proteintech group, China), Ki67 (1 : 2000, 27309-1-AP, Proteintech Group, China), MMP2 (1 : 100, 10373-2-AP, Proteintech Group, China), E-cadherin (1 : 500, 20874-1-AP, Proteintech Group, China), and vimentin (1 : 2500, 10366-1-AP, Proteintech Group, China) at 4°C overnight. Slices were washed thrice with PBS and exposed to the corresponding secondary antibodies for 1 h at room temperature. DAB was used to develop the color for 5 min, and nuclei were restained with hematoxylin for 5 min. Ten randomly selected microscopic areas from each slide were observed by two independent pathologists to record the degree of positive staining and assess the percentage of positive cells, and results were averaged.

### 2.22. Western Blot Analysis

Tumor tissues or cells were lysed on ice with RIPA buffer supplemented with the protease inhibitor PMSF for 20 min to extract the total protein. The protein concentration of each group of samples was determined thrice using the BCA method. The protein from each group (15–30 *μ*g) was separated by SDS-PAGE and transferred into PVDF membranes (EMD Millipore, USA). After being blocked with 5% milk for 2 h, membranes were incubated overnight with primary antibodies: anti-*β*-actin (1 : 1000, cat. no. 4970, Cell Signaling Technology), anti-GAPDH (1 : 1000, cat. no. 5174, Cell Signaling Technology), anti-HO-1 (1 : 1000, ab13243, Abcam, USA), anti-GPX4 (1 : 1000, ab125066, Abcam, USA), anti-FTH1 (1 : 1000, BM4487, Boster Biological Technology, China), anti-FTL/Ferritin Light Chain (1 : 1000, 10727-1-AP, Proteintech Group, China), anti-SLC7A11/XCT (1 : 1000, 26864-1-AP, Proteintech Group, China), anti-SLC40A1/FPN1 (1 : 1000, 26601-1-AP, Proteintech Group, China), anti-DMT1 (1 : 1000, 20507-1-AP, Proteintech Group, China), anti-SOD2 (1 : 1000, 66474-1-Ig, Proteintech Group, China), anti-MMP2 (1 : 1000, 10373-2-AP, Proteintech Group, China), anti-E-cadherin (1 : 1000, 20874-1-AP, Proteintech Group, China), anti-vimentin (1 : 1000, 10366-1-AP, Proteintech Group, China), anti-NRF2 (1 : 1000, 16396-1-AP, Proteintech Group, China), and anti-KEAP1 (1 : 1000, 10503-2-AP, Proteintech Group, China). PVDF membranes were incubated with secondary antibodies for 90 min the next day and visualized with an enhanced chemiluminescence analysis kit (Biosharp, China) on the ChemiDoc MP imaging system (Bio-Rad, USA). All target proteins were quantified and analyzed using the ImageJ software.

### 2.23. Bioinformatics Analysis

All tumor samples in The Cancer Genome Atlas (TCGA, http://cancergenome.nih.gov) and the corresponding normal tissue samples in the Genotype-Tissue Expression (GTEx, https://gtexportal.org/) database were downloaded to analyze the differential expression of HMOX1 in 33 tumors by using the Gene Expression Profiling Interactive Analysis (GEPIA; http://gepia.cancer-pku.cn) database (default parameters: |log_2_FC|cutoff = 1, *q* value cutoff = 0.01). The KIRC dataset included data from 523 tumor and 100 normal control tissues. The HO-1 expression-based survival curves were applied to investigate the effect of HO-1 expression on the survival and prognosis of patients with ccRCC. The overall survival analysis was performed using the Kaplan–Meier analysis, and the log-rank test was applied to calculate the *P* value.

### 2.24. Molecular Docking Technology

The initial structures of HO-1 were collected from the PDB code of 6EHA. The Lut substrate was docked into the active site of protein by using the AutoDock Vina tool (1) in Chimera (2). The docked poses with the highest docking scores were used for subsequent analysis [29, 30].

### 2.25. Statistical Analysis

All experimental data were presented as mean ± SD, and the SPSS 26.0 statistical software and Microsoft Excel 2016 were used for calculation and statistical analysis. For comparison between two groups, Student's *t*-test was used to calculate the *P* value for the significant *P* values of expression differences. Statistical analysis was performed using one-way ANOVA to compare more than two groups, and Tukey's post hoc test was used for pairwise comparisons after one-way ANOVA. Differences with *P* value < 0.05 were considered statistically significant. Graphs were constructed using the GraphPad Prism 8.0 software. All experiments were performed at least thrice.

## 3. Results

### 3.1. Lut Suppresses the Proliferation, Migration, and Invasion of ccRCC Cells

The CCK8 assay showed dose- and time-dependent decreases in cell viability after incubation of 786-O and OS-RC-2 cells treated with 0, 0.5, 1, 2, 4, 8, 16, 32, 64, and 128 *μ*M Lut for 24 or 48 h (Figures 1(b) and 1(c)). The IC50 values of Lut at 24 h were 44.89 and 60.22 *μ*M in 786-O and OS-RC-2 cells, respectively. Therefore, 40 and 60 *μ*M were selected as appropriate concentrations of Lut for 786-O and OS-RC-2 cells, respectively, in subsequent experiments. Microscopy revealed that ccRCC cells elongated into a shuttle shape (786-O) or turned wrinkled and rounded (OS-RC-2) and became slower to proliferate after treatment with Lut for 24 h compared with the control group (Figure 1(d)). Compared with the NC group, the Lut group had evidently suppressed efficiency and number of colony formation in ccRCC cells (Figures 1(e) and 1(h)). The results of the wound healing assay indicated that Lut treatment evidently reduced the migration rates of 786-O and OS-RC-2 cells compared with the control (Figures 1(f) and 1(i)). Similarly, the invasive ability of ccRCC cells treated with Lut for 24 h was considerably restrained compared with that of the NC group (Figures 1(g) and 1(j)).

### 3.2. Fe^2+^ Accumulation and HO-1 Upregulation Contribute to Lut-Induced Cell Death in ccRCC

Compared with the control group, the Lut-treated group had a stable upregulation of intracellular Fe^2+^ levels in a time-dependent manner (Figure 2(a)). Conversely, the levels of intracellular GSH in the Lut-treated group decreased (Figure 2(b)). Subsequently, to elucidate the role of Fe^2+^ in the ccRCC cell death induced by Lut, we examined the alteration of the cell death ratio by regulating the level of Fe^2+^ on the basis of Lut treatment. 786-O and OS-RC-2 cells were pretreated with 600 *μ*M iron chelator DFP or 500 *μ*M FAC for 2 h before Lut treatment for 24 h. The LDH assay indicated that Lut-induced cell death was considerably attenuated in the presence of DFP, whereas FAC exacerbated the killing effect of Lut on ccRCC cells. Likewise, the pretreatment of ccRCC cells with 10 mM ROS inhibitor NAC or 10 *μ*M ferroptosis inhibitor Fer-1 for 2 h was performed prior to incubation with Lut for 24 h. LDH results revealed that NAC and Fer-1 substantially blocked the killing effect of Lut (Figure 2(c)).

Immunoblotting was performed to examine Lut-induced changes in proteins to verify our speculation. Compared with the NC group, 786-O and OS-RC-2 cells treated with Lut for 24 h had evidently downregulated expression levels of GPX4, SLC7A11, SLC40A1, ferritin (FTH1 and FTL), vimentin, and MMP2. Furthermore, interestingly, we found that the HO-1, DMT1, and E-cadherin expression levels were quite remarkably upregulated and that the KEAP1-NRF2 axis was activated by Lut (Figures 2(d) and 2(e)). The above results revealed that Lut probably facilitated intracellular Fe^2+^ production by upregulating HO-1 expression to trigger ferroptosis in ccRCC eventually.

The GEPIA database based on clinical patient data from TCGA and GTEx showed that the basal expression activity of HO-1 in ccRCC ranked first in pan-cancer (Figure 3(a)). The expression of HO-1 in cancerous tissues of KIRC was considerably upregulated compared with that in normal tissues (Figure 3(b)). The western blot was performed and revealed that the expression levels of HO-1 in three types of ccRCC cells (i.e., A498, 786-O, and OS-RC-2) were increased compared with those in HK-2 cells (Figure 3(c)). Interestingly, the survival analysis revealed that patients with KIRC and high HO-1 expression had a higher overall survival rate compared with those with low HO-1 expression, and this finding was not observed in KIRP and KICH (Figure 3(d)). These data implicated that the low expression of HO-1 in KIRC predicted a poor prognosis, which might be improved by elevating the expression of HO-1 in patients with KIRC.

### 3.3. Lut-Induced Suppression of ccRCC Proliferation and Invasion Can Be Alleviated by Inhibiting Ferroptosis or Buffering Fe^2+^ Accumulation

As shown in the CCK-8 assay, the cell viability of 786-O and OS-RC-2 cells treated with Lut or erastin (30 *μ*M) for 24 h was remarkably reduced compared with that of the control group, but this inhibition of cell viability caused by Lut was rescued by pretreatment with 600 *μ*M DFP or 10 *μ*M Fer-1 to some extent (Figure 4(a)). The morphology of most 786-O cells treated with Lut for 24 h gradually changed from oval to elongated with minimal cell confluence, which was partially reversed by DFP or Fer-1 pretreatment (Figures 4(b) and 4(c)). As demonstrated in Figure 4(d), the DNA replication activity of 786-O cells was notably inhibited by Lut or erastin in comparison with that of the NC group, but this restraint was again blocked partly by Fer-1 or DFP (Figures 4(d) and 4(e)). The invasion capabilities of 786-O and OS-RC-2 cells were also visibly limited by Lut (20 *μ*M, low concentration) or erastin, but the number of invaded cells was increased with DFP or Fer-1 pretreatment, as displayed by the Transwell invasion assay (Figures 4(f) and 4(g)).

### 3.4. Fe^2+^ Accumulation Induced by Lut Leads to Mitochondrial Dysfunction and Ferroptosis in ccRCC

To observe mitochondrial damage, we performed the *δψ*M experiment. The JC-1 in the mitochondria of the NC group existed as JC-1 aggregates with bright red fluorescence and weak green fluorescence. Following the induction of ccRCC cells by Lut or erastin, the mitochondrial membrane potential decreased, and JC-1 was unable to exist as JC-1 aggregates in the inner mitochondrial membrane consistently but as JC-1 monomers for the ratio of red to green fluorescence to notably decline. However, the mitochondrial membrane potential was restored to some extent after the administration of the iron chelator DFP (Figures 5(a) and 5(b)). Transmission electron microscopy revealed that OS-RC-2 cells treated with Lut for 24 h exhibited classical ferroptosis manifestations, i.e., decreased or disappeared mitochondrial cristae and increased mitochondrial membrane density (Figure 5(c)). Similar to the erastin group, 786-O and OS-RC-2 cells treated with Lut had substantially induced ROS generation, whereas the ROS level was apparently decreased to about half of that in the Lut group after cotreatment with Lut and DFP (Figures 5(d) and 5(e)). As shown by the C11 BODIPY staining, 786-O cells treated with erastin presented with bright green fluorescence that represented severe lipid peroxidation, which confirmed the manifestation of ferroptosis. As in the erastin group, Lut evoked a substantial accumulation of lipid peroxides and ultimately triggered ferroptosis. Following the administration of Fer-1 and DFP, Lut-induced lipid peroxidation was suppressed to some degree (Figures 5(f) and 5(g)).

The accumulation of LIP and significant depletion of GSH were prominently induced by Lut or erastin, whereas Fe^2+^ and GSH levels were recovered to some extent in ccRCC cells when cotreated with Fer-1/DFP and Lut (Figures 6(a) and 6(b)). Additionally, as demonstrated by immunofluorescence staining, the expression of GPX4 was evidently decreased in Lut and erastin groups, and this inhibition of GPX4 was considerably obstructed by the chelation of Fe^2+^ or direct suppression of lipid peroxidation. Conversely, the expression of HO-1 in 786-O cells was exceedingly upregulated upon administration of Lut or erastin (Figures 6(c) and 6(d)). Interestingly, the overexpression HO-1 could not be further blocked by Fer-1 or DFP on the basis of Lut administration, validating that HO-1 was located upstream of the Fe^2+^ pool and cascade response of ferroptosis (Figures 6(c) and 6(d)). These changes in the expression levels of GPX4 and HO-1 in 786-O and OS-RC-2 cells were also subsequently verified by western blot. Besides, the alterations in SLC7A11 and SOD2 protein levels in ccRCC cells were generally consistent with GPX4, and these data supported the former results of ROS and lipid peroxidation assays (Figure 6(e)).

### 3.5. Blocking the Excessive Upregulation of HO-1 Inhibits Fe^2+^ Accumulation, Thereby Reversing Lut-Induced Ferroptosis in ccRCC

Heme assay showed that Lut substantially reduced the heme level in ccRCC; however, knockdown of HO-1 with siHO-1 or Znpp significantly restored the heme content (Figure 7(a)). When HO-1 was knocked down, the Lut-induced increase in Fe^2+^ was blocked accordingly, which further confirmed that HO-1 contributed to the accumulation of LIP induced by Lut in ccRCC cells (Figure 7(b)). The apparent restoration of GPX4 and SLC7A11, which were previously downregulated by Lut, occurred in response to the knockdown or inhibition of HO-1 (Figures 7(c) and 7(d)). Finally, we examined the influence of changing HO-1 expression on Lut-induced lipid peroxidation by C11 BODIPY staining. These groups, including Lut, Lut+siNC, and Lut+DMSO, displayed a higher level of lipid peroxidation in 786-O cells. The ratio of red to green fluorescence was remarkably elevated after using siHO-1 or Znpp on the basis of Lut (Figures 7(e) and 7(f)). The above results strongly demonstrated that Lut promoted heme degradation by inducing HO-1 overexpression in ccRCC cells, thereby leading to Fe^2+^ overload and ultimately resulting in lipid peroxidation and ferroptosis.

Based on the structures of docking, Figure 7(g) depicts the binding interactions of Lut with HO-1. Results showed that hydrophobic, H-bond, and other noncovalent interactions had key roles in influencing the binding affinity of complexes. Lut was anchored into a hydrophobic pocket in HO-1 and accommodated well into the active center by a *π*-*π* interaction among the phenyl ring of Phe167 and Phe214, the conjugate structure of the substrate, and a hyperconjugative effect interaction between this conjugate structure with Leu54 and Arg136. Moreover, Lut interacted with Asp170 and Asn210 in HO-1 active sites, forming H-bond networks that were fixed in active sites. In view of these interactions, the binding of substrate to amino acids was tight and deep into the cavity, revealing that small molecules were well suited to receptor-binding pockets. In this docking position, the hydroxyl groups of the substrate and the iron ions of heme approached in a relatively close position, and in the process of combining oxygen with heme iron, such a hydroxyl group stabilized oxygen atoms to a certain extent and promoted the metabolic process of heme (Figure 7(g)).

### 3.6. Ferroptosis Is Implicated in the Anti-ccRCC Mechanisms of Lut In Vivo

OS-RC-2 cells were xenografted into the right dorsum of nude mice to establish a xenograft model of human ccRCC and examine the role and mechanism of Lut on ccRCC *in vivo*. The volume and weight of tumors in the Lut and erastin groups were evidently lower than those in the control group, whereas the tumors in the Lut+DFP and Lut+Znpp groups were larger in volume and weight than those in the Lut group. Compared with the controls, the growth of tumors treated with Lut was substantially inhibited by day 7 and slowed appreciably over the next 8 days (Figures 8(a)–8(c)). Histological examination showed that tumor cells existed in the form of cancer nests with vascular distribution between nests, and cells with a transparent and hollow cytoplasm formed dense glandular vesicles and tubular or cystic structures, which demonstrated the success of model establishment (Figure 8(d)). Additionally, the Fe^2+^ assay showed that Lut, similar to erastin, upregulated Fe^2+^ levels in tumor tissues and that this capability of Lut to activate LIP was partially obstructed by DFP or Znpp (Figure 8(e)). Later, we assayed MDA, the product of lipid peroxidation. The production of MDA was apparently induced by Lut and erastin, whereas the presence of DFP or Znpp reduced the Lut-induced MDA production to some extent (Figure 8(f)). Conversely, GSH depletion was evidently evoked by the intervention of Lut or erastin in comparison with controls, whereas DFP or Znpp rescued GSH levels in tumors to some extent by the appropriate chelation of iron ions and inhibition of HO-1 (Figure 8(g)).

Subsequently, western blot showed that the expression levels of E-cadherin and HO-1 were notably enhanced by Lut or erastin, whereas MMP2, vimentin, GPX4, and SLC7A11 expression levels in tumor tissues treated with Lut or erastin were remarkably inhibited compared with those in the controls. However, the presence of DFP or Znpp could reverse the aforementioned Lut-induced protein expression changes of E-cadherin, MMP2, vimentin, GPX4, and SLC7A11 to some extent. The induction of HO-1 by Lut could be alleviated by Znpp and was not observed to be blocked by DFP (Figures 9(a) and 9(b)). Consistent with western blot, immunohistochemistry revealed that Lut downregulated the expression levels of KI67, MMP2, vimentin, GPX4, and SLC7A11 and upregulated the levels of HO-1 and E-cadherin (Figure 9(c)). Collectively, our experimental data demonstrated that ferroptosis is implicated in the anti-ccRCC mechanisms of Lut *in vivo* (Figure 10).

## 4. Discussion

As one of the most common urological malignancies, the therapy for ccRCC has made outstanding achievements, including the development and application of various targeted therapeutic agents, such as VEGF inhibitors, mTOR inhibitors, and immune checkpoint inhibitors, in recent years [31]. These achievements have substantially enhanced the prognosis of a large number of patients with metastatic or unresectable ccRCC. Unfortunately, insensitivity to radiotherapy and chemotherapy, unavoidable drug resistance, and various adverse effects limit the efficacy of these targeted or immunotherapeutic agents [6]. Therefore, the investigation and development of novel antitumor mechanisms and stabilized drugs are imminent. Excitingly, RCC has been discovered to be sensitive to ferroptosis, a novel form of regulated cell death distinct from apoptosis. Moreover, various compounds of natural origin, such as paclitaxel, hydroxycamptothecin, and homoharringtonine, have become the universally recognized agents of anticancer from the second half of the 20th century to the present due to their broad and prominent biological activities, low cost relative to synthesized anticancer medicines, and novel and unique mechanisms of action [32–34]. Here, we found that Lut, a natural flavonoid extracted from plants, induces antitumor activity in ccRCC. Mechanistically, Lut promotes free Fe^2+^ overload in ccRCC cells by mediating heme degradation via inducing HO-1 overexpression. This phenomenon further provokes mitochondrial dysfunction and lipid peroxidation and ultimately triggers ferroptosis in ccRCC.

The primary mechanism of ferroptosis is the Fenton reaction mediated by Fe^2+^ (LIP) or the action of lipoxygenase, which catalyzes PUFAs highly expressed on the cell membrane and expands the lipid peroxidation reaction. Additionally, ferroptosis is manifested by the inactivation of the regulatory core enzyme GPX4 based on GSH depletion [7, 35]. The fact that the kidney is an important organ in iron metabolism and homeostasis and that the abnormally vigorous metabolic status of tumor cells results in a high requirement for iron shows that ferroptosis is prone to be triggered in RCC. Previously, Yang et al. reported that the Hippo pathway effector TAZ regulates ferroptosis in RCC [36]. Wang et al. demonstrated that SUV39H1 deficiency suppresses ccRCC growth by inducing ferroptosis [13]. Markowitsch et al. revealed that artesunate inhibits the cancer growth of sunitinib-resistant RCC cells through cell cycle arrest and induction of ferroptosis [37].

Previous studies showed that Lut is considered potential therapeutic and preventive agents for cancers due to its potent antitumor activity *in vivo and in vitro*. Ou et al. found that Lut induces apoptosis in ccRCC cells (i.e., 786-O, A498, and ACHN), and this apoptosis is mediated by the downregulation of Akt and the upregulation of apoptosis signal-regulated kinase-1, p38, and c-Jun N-terminal kinase activity probably via protein phosphatase 2A activation [38]. Besides, Lut is recognized as a potential sensitizer of TRAIL in anticancer therapy against human RCC involving Akt and STAT3 inactivation [39]. However, so far evidence on whether ferroptosis is also implicated in the anticancer mechanism of Lut is still absent. Our experimental results indicated that Lut suppresses the proliferation, migration, and invasion of ccRCC cells, tentatively validating the stable efficacy of Lut against ccRCC *in vitro*. Afterwards, a notable upregulation of Fe^2+^ levels and ferroptosis were determined in Lut-treated ccRCC cells. The suppression of ccRCC proliferation and invasion induced by Lut was obviously alleviated by inhibiting ferroptosis or preventing Fe^2+^ accumulation. In addition, Lut induced the imbalance of mitochondrial membrane potential, classical morphological alterations of mitochondrial ferroptosis, generation of ROS, and occurrence of lipid peroxidation in an iron-dependent manner among ccRCC cells. Our preliminary findings provided *in vitro* and *in vivo* evidence supporting the notion that ferroptosis contributes to Lut-induced cell death in ccRCC.

Thereafter, we examined various ferroptosis pathways to probe the potential mechanisms of Lut-triggered ferroptosis. We focused on HO-1 based on experimental results, and surprisingly, a substantial (up to 11.4-fold) and persistent upregulation of HO-1 in response to Lut stimulation, excluding compensatory effects, contradicts our previous recognition of HO-1 (protective factor). HO-1, the essential rate-limiting enzyme of heme metabolism, is previously considered to exert potent cytoprotective functions under various stress conditions. However, latest studies reveal a dual role for HO-1. HO-1 exerts a protective effect by scavenging ROS upon appropriate activation, but when excessively activated, HO-1 can boost the accumulation of LIP, contributing to ROS overload and activating the ferroptosis cascade [26]. Fang et al. demonstrated that HO-1 is upregulated by nuclear translocation of Nrf2 in adriamycin-induced cardiac injury, thereby catalyzing the degradation of heme, promoting the release of free Fe^2+^, and resulting in ferroptosis and ultimately heart failure [25]. Fernández-Mendívil et al. confirmed that the microglial HO-1 overexpression in aged mice exposed to an acute inflammatory insult favors iron accumulation, ferroptosis, and memory impairment [40]. Malfa et al. reported that the *Betula etnensis* Raf. extract promotes an oxidative cellular microenvironment, resulting in human colon cancer cells by ferroptosis mediated by HO-1 hyperexpression [41]. Furthermore, curcumin, tagitinin C, and BAY 11-7085 are identified to result in the occurrence of ferroptosis in various tumors through upregulating HO-1 [42–44]. These recent studies suggested that the excessive upregulation and activation of HO-1 to trigger ferroptosis are probably a promising strategy for oncologic chemotherapy. Coincidentally, bioinformatics analysis revealed that the high expression of HMOX1 predicts a better prognosis for patients with ccRCC. A primary endogenous source of free Fe^2+^ is the enzymatic catabolism of heme via HO-1 [45]. As a ubiquitous protoporphyrin IX ring, heme could serve as a Fenton reactor to generate toxic hydroxyl radicals due to the presence of an individual Fe^2+^ ion in its center [46]. Heme metabolism takes place in all mammalian cells [47]. Through a three-step process requiring oxygen and reducing equivalents from NADPH, protoheme is degraded to equimolar amounts of labile Fe^2+^, carbon monoxide, and biliverdin IX*α* by heme oxygenase-1 [48, 49]. NADPH-cytochrome P450 reductase provides electrons for HO-1 catalysis in mammals [48]. The free Fe^2+^ released from heme is too toxic to remain at large in cells and would be promptly neutralized by Fe metabolic pathways including the induction of an iron efflux pump as well as the induction of ferritin, a Fe sequestering protein, which is the major iron ion storage protein in the cytoplasm (4,500 mol of iron/mol of ferritin) [46, 50, 51]. Consequently, HO-1 could suppress the cytotoxic effects of free heme by mediating heme catabolism under normal conditions. Expression of HO-1 could be regulated at the transcriptional level [46]. Suttner et al. suggested that there exists a beneficial threshold of HO-1 overexpression associated with the accumulation of reactive Fe^2+^ released from the degradation of heme [52]. In response to certain drugs or stimuli, sustained HMOX1 induction degrades heme extensively and leads to the accumulation of labile Fe^2+^, overwhelming the buffering capacity of ferritin. Subsequently, an elevated level of free Fe^2+^ in the iron pool of cells will effectively render the sensitivity of cells to ferroptosis [53]. On the other hand, the elevated Fe^2+^-driven Fenton reaction results in the generation of hydroxyl radical (OH^•^) that stems from H_2_O_2_. Hydroxyl radical can react with LH to engender LOO^•^, while LH also can be oxidized by LOXs to LOOH, which will be further converted into LOO^•^ through the Fenton reaction. Finally, LOO^•^ initiates lipid peroxidation and ferroptosis [54, 55]. Our following experiments further determined that the expression level of HO-1 in ccRCC cells was increased excessively upon Lut treatment accompanied by a noticeable increase in free Fe^2+^ and substantial degradation of heme. Knockdown of HO-1 restored heme levels remarkably and reduced the increased Fe^2+^ almost back to normal levels, which considerably attenuated the degree of lipid peroxidation in ccRCC. The increased iron uptake mediated by overexpressed DMT1, reduced iron efflux due to decreased FPN1, and the Lut-induced downregulation of ferritin may also contribute to free Fe^2+^ overload during ferroptosis. In addition, HO-1-mediated ferroptosis was also implicated in the anti-ccRCC mechanisms of Lut *in vivo*. At last, the molecular docking of Lut with HO-1 indicates that Lut is well suited to the receptor-binding pockets of HO-1, suggesting that Lut probably enhances the expression or improves the activity of HO-1 and most likely facilitates the metabolic process of heme by stabilizing oxygen atoms.

Some limitations remain in our present study. Several studies proposed that NRF2 exerts resistance to ferroptosis by regulating SLC7A11 [56]. By contrast, the data of the current study suggests that Lut activates the NRF2/HO-1 axis in ccRCC and that the deteriorating effect caused by HO-1 overactivity has exceeded the antiferroptosis effect of the NRF2/SLC7A11 axis, ultimately accounting for the downregulation of SLC7A11 and initiation of ferroptosis. The differences of this effect may be closely associated with the dual function of HO-1, particular drug activities, and various disease models. The mechanism of ferroptosis in ccRCC is extremely complex and not yet well understood, and the complicated metabolism in tumor cells makes ferroptosis elusive. However, the present study shows that the role of HO-1 and the mechanisms of Lut and HO-1 in ferroptosis in ccRCC need to be further investigated. The validation of our current findings with other ccRCC cell lines is still needed. The localization of Fe^2+^ in the organelles in ccRCC cells is of great relevance and deserves to be further investigated. Finally, whether Lut can be utilized as a clinical anticancer agent remains unclear, and extensive and large-scale clinical trials and follow-up studies are necessary.

## 5. Conclusion

In conclusion, our results demonstrate that Lut triggers ferroptosis in ccRCC by excessively upregulating HO-1 expression and activating LIP, thereby exerting antitumor effects. These findings indicate that Lut is a potential inducer of ferroptosis and probably holds potential for application in adjuvant chemotherapy for ccRCC.

## Figures and Tables

**Figure 1:** Lut inhibited ccRCC proliferation, migration, and invasion *in vitro.* (a) Chemical structure of luteolin. CCK-8 assay showed that Lut inhibited the viabilities of 786-O (b) and OS-RC-2 (c) cells in a dosage- and time-dependent manner. (d) Morphological changes of 786-O and OS-RC-2 cells treated with or without Lut for 24 h (magnification, ×40). (e) The colony formation assay of 786-O and OS-RC-2 cells treated with or without Lut for 14 days. (f) The wound healing assay of 786-O and OS-RC-2 cells treated with or without Lut for 24 h (magnification, ×40). (g) Transwell invasion assay of 786-O and OS-RC-2 cells treated with or without Lut for 24 h (magnification, ×200). Semiquantification of colony formation assay (h), wound healing assay (i), and Transwell invasion assay (j). The data in (h), (i), and (j) are expressed as the mean ± SD. ^∗^*P* < 0.05 vs. the NC group. NC: negative control; Lut: luteolin.

**Figure 2:** The accumulation of Fe^2+^ and upregulation of HO-1 are involved in Lut-induced cell death in ccRCC. Levels of intracellular ferrous Fe^2+^ (a) and GSH (b) of 786-O and OS-RC-2 cells treated with or without Lut for 24 h or 48 h. (c) The LDH release assay showed that Lut-induced cell death of ccRCC was alleviated in the presence of DFP, NAC, and Fer-1 and was exacerbated in the presence of FAC. (d) Expression levels of MMP2, vimentin, E-cadherin, HO-1, KEAP1, NRF2, GPX4, SLC7A11, SLC40A1, DMT1, FTL, and FTH1 in 786-O and OS-RC-2 cells treated with or without Lut for 24 h as determined by western blot analysis. (e) Semiquantification of band densities in (d). The data in (a), (b), (c), and (e) are expressed as the mean ± SD. ^∗^*P* < 0.05 vs. the NC group, ^#^*P* < 0.05 vs. Lut group. Lut: luteolin; DFP: deferiprone; NAC: acetylcysteine; Fer-1: ferrostatin-1; FAC: ammonium iron (III) citrate.

**Figure 3:** HMOX1 (HO-1) expression was significantly upregulated in KIRC, and its low expression predicted a poor prognosis. (a) HMOX1 expression profile across all tumor samples and paired normal tissues based on TCGA and GTEx database. (b) The expression of HMOX1 was significantly upregulated in KIRC compared to normal tissue. (c) Expression levels of HO-1 in A498, OS-RC-2, and 786-O cells as determined by western blot analysis. (d) Low expression of HMOX1 in KIRC predicted a poor prognosis (not in KIRP and KICH) with statistically significant significance. The data in (c) are expressed as the mean ± SD. ^∗^*P* < 0.05 vs. the normal tissue group, ^#^*P* < 0.05 vs. HK-2 group. TCGA: The Cancer Genome Atlas; GTEx: Genotype-Tissue Expression; KIRC: kidney renal clear cell carcinoma; KIRP: kidney renal papillary cell carcinoma; KICH: kidney chromophobe.

**Figure 4:** Suppression of ferroptosis and buffering of Fe^2+^ accumulation alleviate proliferation inhibition and invasion inhibition of ccRCC induced by Lut. (a) Results of the CCK-8 assay in 786-O and OS-RC-2 cells, respectively. (b) Morphological changes of 786-O cells treated under different conditions (magnification, ×40). (c) Phalloidin staining of 786-O cells treated under different conditions (magnification, ×400). (d) Proliferative ability of 786-O cells treated under different conditions displayed by the EdU assay (magnification, ×200). (e) Semiquantification of EDU in (d). Representative images (f) and semiquantitative analyses (g) of 786-O and OS-RC-2 cells according to Transwell invasion assays (magnification, ×200). The data in (a), (e), and (g) are expressed as the mean ± SD. ^∗^*P* < 0.05 vs. the NC group, ^#^*P* < 0.05 vs. Lut group. EdU: 5-ethynyl-2′-deoxyuridine; Lut: luteolin; DFP: deferiprone; Fer-1: ferrostatin-1.

**Figure 5:** Lut significantly promotes mitochondrial dysfunction and lipid peroxidation in an iron-dependent manner. Representative images (a) and semiquantitative analyses (b) of JC-1 fluorescence in 786-O cells treated under different conditions (magnification, ×200). (c) Transmission electron microscopy (TEM) observation of mitochondria in OS-RC-2 cells. Representative images (d) and semiquantitative analyses (e) of ROS in 786-O and OS-RC-2 cells treated under different conditions (magnification, ×200). Representative images (f) and semiquantitative analyses (g) of lipid peroxidant in 786-O cells treated under different conditions (magnification, ×200). The data in (b), (e), and (g) are expressed as the mean ± SD. ^∗^*P* < 0.05 vs. the NC group, ^#^*P* < 0.05 vs. Lut group. ROS: reactive oxygen species; Lut: luteolin; DFP: deferiprone; Fer-1: ferrostatin-1.

**Figure 6:** HO-1 overexpression and Fe^2+^ accumulation were implicated in Lut-induced ferroptosis in ccRCC. Levels of intracellular ferrous ion (a) and GSH (b) of 786-O and OS-RC-2 cells treated under different conditions. (c) The expression of GPX4 and HO-1 in 786-O cells treated under different conditions as determined by immunofluorescence staining (magnification, ×400). (d) Semiquantification of GPX4 and HO-1 expression levels in (c). (e) Expression levels of HO-1, GPX4, SLC7A11, and SOD2 in 786-O and OS-RC-2 cells treated under different conditions as determined by western blot. The data in (a), (b), (d), and (e) are expressed as the mean ± SD. ^∗^*P* < 0.05 vs. the NC group, ^#^*P* < 0.05 vs. Lut group. Lut: luteolin; DFP: deferiprone; Fer-1: ferrostatin-1.

**Figure 7:** Silencing or inhibition of HO-1 in an appropriate range can reverse Lut-induced ferroptosis in ccRCC by restraining Fe^2+^ production. (a) Heme levels in 786-O cells treated under different conditions. (b) Levels of intracellular ferrous ion of 786-O cells treated under different conditions. (c) Expression levels of HO-1, GPX4, and SLC7A11 in 786-O cells treated under different conditions as determined by western blot. (d) Semiquantification of band densities in (c). Representative images (e) and semiquantitative analyses (f) of lipid peroxidant in 786-O cells treated under different conditions (magnification, ×200). (g) Interactions of Lut with HO-1 as predicted by molecular docking technology. The data in (a), (b), (d), and (f) are expressed as the mean ± SD. ^∗^*P* < 0.05 vs. the NC group, ^#^*P* < 0.05 vs. Lut+siNC group, and ^&^*P* < 0.05 vs. Lut+DMSO group. Lut: luteolin; Znpp: zinc protoporphyrin.

**Figure 8:** Therapeutic effects of Lut against OS-RC-2 ccRCC xenografts. (a) Representative image of OS-RC-2 xenograft tumors under different treatments. (b) Tumor volume in each group. (c) Weight of xenograft tumors in each group. (d) Representative H&E-stained images of xenograft tumors in each group (magnification, ×400). Levels of Fe^2+^ (e), GSH (f), and MDA (g) of xenograft tumors in each group. The data in (b), (c), (e), (f), and (g) are expressed as the mean ± SD. ^∗^*P* < 0.05 vs. the NC group, ^#^*P* < 0.05 vs. Lut group. Lut: luteolin; DFP: deferiprone; Znpp: zinc protoporphyrin; MDA: malondialdehyde.

**Figure 9:** Ferroptosis is implicated in the anti-ccRCC mechanisms of Lut *in vivo*. (a) Expression levels of E-cadherin, MMP2, vimentin, HO-1, and GPX4 of xenograft tumors in each group as determined by western blot. (b) Semiquantitative analyses of band densities in (a). (c) Expression and semiquantification of KI67, E-cadherin, MMP2, vimentin, HO-1, SLC7A11, and GPX4 in xenograft tumors were analyzed by immunohistochemistry (magnification, ×400). The data in (b) and (c) are expressed as the mean ± SD. ^∗^*P* < 0.05 vs. the NC group, ^#^*P* < 0.05 vs. Lut group. Lut: luteolin; DFP: deferiprone; Znpp: zinc protoporphyrin.

**Figure 10:** A schematic diagram illustrating the mechanism by which HO-1 contributes to luteolin-triggered ferroptosis in clear cell renal cell carcinoma via increasing the labile iron pool and promoting lipid peroxidation.

## Data Availability

*Bioinformatics Analysis*. All tumor samples in The Cancer Genome Atlas (TCGA, http://cancergenome.nih.gov) and the corresponding normal tissue samples in the Genotype-Tissue Expression (GTEx, https://gtexportal.org/) database were downloaded to analyze the differential expression of HMOX1 in 33 tumors by using the Gene Expression Profiling Interactive Analysis (GEPIA; http://gepia.cancer-pku.cn) database (default parameters: |log_2_FC|cutoff = 1, *q* value cutoff = 0.01). The KIRC dataset included data from 523 tumor and 100 normal control tissues. The HO-1 expression-based survival curves were applied to investigate the effect of HO-1 expression on the survival and prognosis of patients with ccRCC. The overall survival analysis was performed using the Kaplan–Meier analysis, and the log-rank test was applied to calculate the *P* value. *Molecular Docking Technology*. The initial structures of HO-1 were collected from the PDB code of 6EHA. The Lut substrate was docked into the active site of protein by using the AutoDock Vina tool (1) in Chimera (2). The docked poses with the highest docking scores were used for subsequent analysis.
